# Shenxian-Shengmai Oral Liquid Evoke Autophagy of Fibroblast to Attenuate Sinoatrial Node Fibrosis in Sick Sinus Syndrome Mice via the AKT/mTOR Pathway

**DOI:** 10.1155/2022/5219277

**Published:** 2022-09-28

**Authors:** Chen Chen, Heng Zhang, Siyi Hou, Yue Liu, Lu Ren, Miao Hao, Keyan Chen, Lingkang Li, Xintong Cai, Zisu Deng, Zhuang Liu, Ping Hou

**Affiliations:** ^1^Liaoning University of Traditional Chinese Medicine, Shenyang, China; ^2^Department of Cardiology, Affiliated Hospital of Liaoning University of Traditional Chinese Medicine, Shenyang, China; ^3^Department of Laboratory Animal Science, China Medical University, Shenyang, China

## Abstract

Sick sinus syndrome (SSS) is closely associated with cardiac syncope and sudden death, wherein sinoatrial node (SAN) fibrosis is one of the main pathological changes that occur. Shenxian-Shengmai oral liquid (SXSM) has been clinically proven to significantly improve the heart rate of SSS patients. In this study, we aimed to explore the mechanism of SXSM in reducing the SAN fibrosis by combining *in vitro* and *in vivo* experiments. Accordingly, the SSS model was constructed by slowly pumping angiotensin II (AngII) with a micro-osmotic pump. The degree of fibrosis was evaluated by Masson's trichrome staining and immunofluorescence staining of the fibrosis marker protein. In addition, NIH-3T3 mouse fibroblasts were used to simulate SAN fibroblasts to further explore the mechanism, with AngII used as the cellular fibrosis inducer. Monodansylcadaverine (MDC) staining and transmission electron microscopy were employed to assay the autophagy content, whereas immunofluorescence staining and Western blotting were employed to elucidate the related protein expression. Finally, fibroblasts were given the AKT phosphorylation agonist SC79 to reversely verify the effects of SXSM. The results showed that SXSM could significantly increase the heart rate of SSS mice by reducing the deposition of extracellular matrix (ECM) in SAN induced by AngII. According to *in vivo* experiments, when compared with the model group, SSS mice treated with SXSM developed less fibrosis in the SAN area. *In vitro* experiments revealed that AngII could restrain autophagy by activating the phosphorylation of the AKT/mTOR pathway, thereby increasing the deposition of ECM. Moreover, SXSM pretreatment prevented this upregulation. After the intervention of SC79, the protective effect of SXSM was weakened. In conclusion, SXSM activated autophagy through the AKT/mTOR pathway, which in turn reduced the deposition of the ECM in SAN induced by AngII, attenuated the fibrosis of SAN, and improved the decreased heart rate in the SSS mice.

## 1. Introduction

Sick sinus syndrome (SSS) is a clinical syndrome of various arrhythmias caused by sinoatrial node (SAN) abnormal pacing or conduction dysfunction. The clinical spectrum of the disorder includes chronotropic incompetence, periodic sinus bradycardia, and paroxysmal sinus pause [1], which is one of the common causes of cardiogenic syncope and sudden death [2]. Although SSS is associated with a high incidence rate and high harm, its effective treatment is limited to artificial cardiac pacemaker implantation. Moreover, no guideline and consensus recommendation has so far been established for long-term tolerable drugs. Intravenous atropine and *β*-adrenergic agonist have been deemed effective for a short time, but long-term application has been reported to result in cardiotoxicity and ventricular arrhythmia [3]. Owing to technical, economical, and artificial factors, the application rate of artificial cardiac pacemaker implantation that is effective for the treatment of SSS is extremely low. Meanwhile, artificial cardiac pacemaker implantation offers the disadvantages of high cost and several contraindications, which may be accompanied by complications such as infection or bleeding in case of implantation or replacement [4]. Biological pacing is still at its basic research stage, and hence there is an urgent need for effective and long-term tolerated drugs for SSS treatment.

Shenxian-Shengmai oral liquid (SXSM) was introduced to the market in 2008. This Chinese patent medicine has been clinically validated over more than 10 years in significantly improving the heart rate and is widely used for the treatment of bradyarrhythmia [5]. The main ingredients of SXSM are *ginseng*, *wolfberry*, *epimedium*, *psoralen*, *salvia*, *ephedra*, *asarum*, and leech. Owing to its remarkable curative effect and long-term tolerability, it offers a broad application prospect in the field of SSS treatment.

The pathogenesis of SSS may be related to the destruction of the connection between myocardial cells by collagen fiber bundles in the process of SAN fibrosis, which in turn leads to slow conduction or discontinuous conduction. Meanwhile, the change in the ion flow caused by the coupling of fibroblasts with myocardial cells also has some effect [6]. As one of the endogenous causes of SSS, the process of fibrosis is closely related to an increase in the angiotensin II (AngII) secretion caused by the activation of the Renin-Angiotensin-Aldosterone System (RAAS) system. AngII can mediate the fibrosis and apoptosis of SAN cells in this process [7, 8]. Degenerative fibrosis of the SAN caused by aging is a common cause of SSS [9]. The pathological changes of fibrosis mainly involve the activation of fibroblasts and the excessive secretion of extracellular matrix (ECM), and the transformation of fibroblasts into myofibroblasts of their activated phenotype is the key event in this process [10, 11]. The activation of fibroblasts significantly expresses alpha-smooth muscle (*α*-SMA) and produces excessive ECM, including fibronectin and collagen-I [10].

Autophagy is a highly conservative programmed degradation mechanism that mostly occurs under the condition of nutritional deficiency or cell stress. Not only is autophagy extremely important for normal cell survival but it also plays an important role in maintaining the homeostasis of the intracellular environment and regulating cell differentiation [12]. Autophagy is mainly manifested in the formation of autophagosomes by double-membrane vesicles and cargo proteins, followed by fusion with lysosomes to digest contents so as to provide energy for cells and renew the cells. This process is regulated by autophagy-related (Atg) protein, Beclin-1, and microtubule-associated protein light-chain 3B (LC3B). In the process of autophagy, Benlin1 is the key protein of autophagy initiation and it participates in the construction of autophagosomes [13]. The microtubule-associated protein light-chain 3B is a marker protein existing on the membrane surface of autophagosomes, including LC3-I and LC3-II. The transformation from LC3-I to LC3-II is the key step in autophagosomes formation. Simultaneously, p62 was used as a substrate to combine with LC3-II, and the complex was finally degraded by lysosome [14, 15]. The occurrence of several heart diseases was related to the change in the autophagy level, including myocardial ischemia-reperfusion injury, myocardial infarction, heart failure, and myocardial hypertrophy [16]. Some past studies have demonstrated that excessive cardiac pressure load can lead to increased myocardial protein synthesis, myocardial fibrosis, and myocardial hypertrophy, accompanied by a decrease in the autophagy activity of cardiomyocytes [17]. Several types of signaling pathways regulate autophagy to an extent. It has been proven that the AKT/mTOR signal pathway is an important regulatory mechanism of autophagy and that it participates in the baseline regulation of autophagy and the regulation during stress [18, 19]. mTOR is a serine/threonine-protein kinase belonging to the phosphatidylinositol kinase-related kinase (PIKK) family. As the key factor of autophagy regulation, mTOR mainly forms two complexes, rapamycin-sensitive complex 1 (mTORC1) and rapamycin-insensitive complex 2 (mTORC2), among which mTORC1 is most closely related to autophagy regulation. mTORC1 participates in the regulation of transcription and the translation of autophagy-related genes by regulating the downstream signaling factors 4E-binding protein 1 (4E-BP1) and ribosomal protein S6 kinase 1 (S6K1) [20, 21].

SXSM has been clinically demonstrated to exert a clear heart rate-enhancing effect, including several Chinese medicines such as *ginseng*, *ephedra*, *epimedium*, *salvia*, and leech. Its effective components, ginsenoside Rh2, icariin, tanshinone IIA, and leech extract possess anti-fibrosis properties [22–26]. However, it is unclear whether it can attenuate the SAN fibrosis of SSS. Therefore, the present study aimed to explore whether it can attenuate the SAN fibrosis of SSS and its mechanism so as to provide further evidence supporting SXSM for its use in the treatment of SSS. During this research, we used AngII to build a mice SSS model and explore the intervention effects of SXSM. In the cell experiments, NIH-3T3 mouse fibroblasts were used to simulate SAN fibrosis toward further exploring the fibrosis-improving mechanism of SXSM [27].

## 2. Methods and Materials

### 2.1. Animal Study

All experimental mice in this research were purchased from Liaoning Changsheng Biotechnology [China, production license SCXK (Liao) 2018–0001] and adaptively raised as per the guidelines of the Experimental Animal Center of China Medical University for 1 week. A total of 15 mice (male or female) were randomly assigned to 3 groups: sham-operation group (SHAM, *n* = 5), SSS model group constructed by AngII (SSS, *n* = 5), and SXSM treatment group (SXSM, *n* = 5). The experiment was performed as per the method described by Swaminathan et al. [28]. Briefly, the mice fasted for 24 h before modeling, and then the SSS model was established through subcutaneously pumping AngII (3 mg/kg/day) with a micro-osmotic pump (Alzet model 1004, 0.11 *μ*/h, 30 days). The specific construction method used was as follows: before the operation, an Alzet osmotic capsule was placed at 37°C in normal saline for 6 h for activation. After the mouse neck-skin preparation, 1% pentobarbital sodium (45 mg/kg) was injected intraperitoneally for anesthesia, and the mice were fixed on an animal operating table in the prone position. Then, a 1–1.5 cm incision was created in the neck to prepare a pouch and the activated micro-osmotic pump was loaded with AngII. The micro-osmotic pump loaded with normal saline was placed in the CON group. Then, all the mice were administered a small amount of gentamicin to prevent postsuture infection. On the second day of operation, the drug was administered via gavage. The SXSM group was provided with the SXSM (Buchang Pharma, China) (5 mL/kg/days), and the other experiment groups received the same amount of pure water. After 30 days, the heart rates of the mice were recorded and analyzed with an electrocardiogram. After euthanasia with 1% pentobarbital sodium (150 mg/kg), the heart tissues of the mice were immediately collected and fixed in 4% paraformaldehyde.

### 2.2. Masson's Trichrome Staining

The heart tissues were sliced in 5-*μ*m transverse sections after paraffin embedding. Then, these paraffin sections were dewaxed and washed with distilled water. The nuclei were stained with Weigert's iron hematoxylin, rinsed with distilled water, and then stained in Masson's composite staining solution for 5 min. The sections were soaked in 1% glacial acetic acid solution and then differentiated with 1% phosphomolybdic acid buffer for 5 min. Without washing, the slices were counterstained with aniline blue for 5 min and then washed with the 0.2% glacial acetic acid solution. Finally, 95% ethanol and absolute ethanol were used to dehydrate the slices, and the neutral gum was sealed after cleaning in xylene. The SAN area of the slices was observed under an optical microscope, and the collagen volume fraction in this area was statistically analyzed to evaluate the degree of SAN fibrosis.

### 2.3. Cell Culture

NIH-3T3 mouse fibroblasts were purchased from ATCC (USA). The cells were inoculated into a cell culture dish and cultured in a medium composed of 89% DMEM/F12 (Hyclone, USA) supplemented with 10% fetal bovine serum (Sijiqing, China) and 1% penicillin/streptomycin (Procell, China). Cell culture was conducted in an incubator containing 5% CO_2_ at 37°C.

The cultured cells were categorized into four groups: CON, AngII, SXSM, and SC79. CON was used as a blank control group without any intervention measurements. The cells in the other groups were treated with AngII (Sigma-Aldrich, USA) for 48 h after culturing for 12 h, while the SXSM group was treated with SXSM, and the SC79 group was treated with SXSM in combination with the AKT phosphorylation agonist SC79 (Topscience, China). The concentration of AngII was 0.1 *μ*M, and those of SXSM and SC79 were 1 mL/L and 8 *μ*g/mL, respectively. The optimal concentration of SXSM was obtained by cell viability testing.

### 2.4. Cell Viability Assay

NIH-3T3 cells (100 *μ*L) were inoculated into a 96-well plate at the density of 1 × 10^4^ cells/mL and categorized into 6 groups. Meanwhile, each group was assigned 5 additional wells. After 12 h of culturing, each group received different concentrations of SXSM (0, 0.5, 1, 2, 5, and 10 mL/L), and the medium was removed after 12, 24, and 48 h. Finally, the cell count kit 8 (CCK-8) (Apex Biotechnology, USA) was used to measure the cell viability.

### 2.5. Immunofluorescence Staining

*In vivo* experiments, the paraffin sections of the SAN tissues were dewaxed and dehydrated and then sealed with 1% BSA for 1 h. After sealing, fibronectin and collagen-I antibodies were added, and the sections were placed overnight in a wet box at 4°C. After washing the sections with PBS, the second antibody labeled with CoraLite488 fluorescein was added and incubated at 37°C for 1 h. After washing again, the antifluorescence quenching solution containing DAPI was added. Finally, the sections were observed under a fluorescence microscope. In *in vitro* experiments, NIH-3T3 cells (1 mL) were inoculated into a confocal dish at the density of 1 × 10^4^ cells/mL. After the abovementioned culture and treatment, 4% paraformaldehyde was added and the cells were fixed for 20 min and then permeabilized with an immune permeabilization solution for 20 min. After washing with PBS, the cells were blocked in 1% BSA for 1 h, followed by the addition of the primary antibody and incubated in a damp box at 4°C overnight. After washing with PBS, the second antibody labeled with the CoraLite488 fluorescein was added and incubated at 37°C for 1 h. Finally, after washing again with PBS, the cells were treated with an antifluorescence quenching mounting tablet containing DAPI and observed under a laser scanning confocal microscope. The collagen-I primary antibody, fibronectin primary antibody, and CoraLite488-conjugated affinipure goat antirabbit IgG were purchased from Proteintech (China).

### 2.6. Monodansylcadaverine Staining

The autophagy rate of cells was detected by MDC staining. NIH-3T3 cells were suspended after digestion in the trypsin–EDTA solution, washed with a wash buffer, and resuspended again, followed by staining with the MDC staining solution at 37°C for 30 min. After washing with the wash buffer, the cells were resuspended in a collection buffer and then detected by flow cytometry. The MDC kit was purchased from Solarbio Biotechnology (China).

### 2.7. Transmission Electron Microscopy

NIH/3T3 cells were inoculated in dishes for the abovementioned culture and treatment processes. After digesting with the trypsin–EDTA solution, the cells were collected via centrifugation at 1200 rpm for 10 min, and 2.5% glutaraldehyde was added for fixation at 4°C for 2 h. After washing with phosphate buffer, 1% osmic acid was added for fixation at 4°C for 1 h and then washed with phosphate buffer. The cells were embedded after dehydration with the gradient dehydration method and then placed on an ultramicrotome to prepare ultrathin sections of 50–70-nm thickness. Finally, the sections were stained with uranus acetate and lead citrate and then observed by transmission electron microscopy.

### 2.8. Western Blotting

NIH/3T3 cells were cultured and treated as described above. After protein extraction, the target protein was quantified by the BCA protein assay kit (Wanleibio, China), heated at 100°C for 5 min to denature, and stored at −20°C. The protein was separated in 10% sodium dodecyl sulfate-polyacrylamide gel (SDS-PAGE) (Wanleibio, China) and then transferred onto a 0.45-*μ*m PVDF membrane via electrophoresis in Tris-glycine buffer (Solarbio Biotechnology, China). The PVDF membrane was blocked in Tris-buffered saline containing 0.05% Tween-20 (TBST) with 5% skimmed milk powder at room temperature for 1 h, followed by incubation with AKT, p-AKT, mTOR, p-mTOR, GAPDH, Beclin-1, p62, LC3-I, and LC3-II primary antibodies for overnight at 4°C. Then, the PVDF membrane was washed with TBST and incubated with a secondary antibody at room temperature for 1 h. Finally, after washing with TBST, the membrane was exposed and imaged using the ECL chemiluminescence kit (Beyotime, China). HRP-conjugated affinipure goat antirabbit IgG was sourced from Wanleibio (China).

### 2.9. Statistical Analysis

The experiment was repeated thrice, and the experimental data at all three times were statistically analyzed by SPSS 25 and expressed as the mean ± SD. One-way analysis of variance (ANOVA) was applied to conduct comparison among the groups, with *P* < 0.05 considered to indicate statistical significance.

## 3. Results

### 3.1. Shenxian-Shengmai can Improve the Sinus Node Function by Improving Angiotensin II-Induced Sinus Node Fibrosis

The heart rate and the ECG R-R interval of each group were used to evaluate the function of the SAN in mice. Masson's trichrome staining and immunofluorescence staining of the fibrosis marker protein were performed to evaluate the degree of SAN fibrosis in mice. Electrocardiogram revealed that the heart rate of the SSS group mice decreased significantly, while the R-R interval was prolonged, suggesting that AngII could successfully induce SSS. Meanwhile, the heart rate and the R-R interval of the mice in the SXSM group were significantly improved (Figures 1(a)–1(c)). Masson's trichrome staining and immunofluorescence staining results revealed that, when compared with the SHAM group, the degree of fibrosis in the SSS group increased significantly under the induction of AngII, accompanied by a significant expression of fibrotic proteins, such as fibronectin and collagen-I. When compared with the SSS group, the degree of fibrosis and the expression of the fibrotic protein in the SXSM group were significantly improved (Figures 2(a) and 2(b)). Statistical analysis of the collagen volume fraction and average optical density in the SAN area of mice from each group indicated that SXSM significantly resisted the fibrosis of the SAN area induced by AngII (Figures 2(c) and 2(d)). In summary, SXSM could significantly attenuate SAN fibrosis induced by AngII, thereby improving the function of the SAN.

### 3.2. Optimum Concentration Screening of SXSM

No cytotoxicity was observed in Shenxian-Shengmai treatment at a concentration of 0–10 ml/L for 12–48 h. The activity of NIH-3T3 cell line under the action of different concentrations of SXSM was analyzed by CCK-8. The cell viability was considered to be 100% when pretreated with SXSM at the concentration of 0 mL/L. No cytotoxicity was recorded in the NIH-3T3 cell lines treated with different concentrations of SXSM for 12, 24, and 48 h, with the maximum effect recorded at 1 mL/L (Figure 3). The following experiments were performed under the condition of 1 mL/L of SXSM treatment for 48 h. We noted that the viability of NIH-3T3 cells was the best under these conditions.

### 3.3. SXSM Reduced Fibrosis of NIH-3T3 Cell Line

The expression of *α*-SMA, fibronectin, and collagen-I in the NIH-3T3 cell line was detected by immunofluorescence staining to evaluate the degree of cell fibrosis. The results indicated that, when compared with the CON group, the fluorescence intensity of *α*-SMA, fibronectin, and collagen-I in NIH-3T3 cells treated with AngII increased significantly. Meanwhile, when compared with the AngII group, SXSM improved the overexpression of *α*-SMA, fibronectin, and collagen-I in NIH-3T3 cells induced by AngII; however, this improvement of SXSM could be blocked by AKT phosphorylation agonist SC79 (Figures 4(a)–4(d)). Thus, we concluded that SXSM can resist NIH-3T3 fibroblast fibrosis by attenuating AKT phosphorylation.

### 3.4. SXSM Activates Autophagy of NIH-3T3 Fibroblasts

The autophagy level of NIH-3T3 fibroblasts was evaluated by MDC staining, and the number of autophagosomes was determined by transmission electron microscopy. The results of MDC staining revealed that the autophagy level of NIH-3T3 cells treated with AngII decreased significantly. When compared with NIH-3T3 cells induced by AngII, the autophagy rate of NIH-3T3 cells induced by AngII treated with SXSM increased significantly. Notably, the activation of SXSM on autophagy could be blocked by AKT phosphorylation agonist SC79 (Figures 5(a) and 5(c)). The results of transmission electron microscopy revealed that the number of autophagosomes in NIH-3T3 cells induced with AngII decreased significantly. On the other hand, the number of autophagosomes in NIH-3T3 cells induced with AngII increased significantly in the presence of SXSM; this trend was reversed after the addition of SC79 (Figures 5(b) and 5(d)). This result was consistent with the results of MDC staining. In summary, we concluded that the activation of SXSM on autophagy of NIH-3T3 fibroblasts may have been caused through the activation of AKT phosphorylation.

### 3.5. Protein Assay of the Akt/mTOR Signaling Pathway and Autophagy

Beclin-1, p62, LC3-I, and LC3-II are the signature proteins of autophagy, and their expressions are closely related to the phosphorylation level of the AKT/mTOR signaling pathway. Therefore, we employed Western blotting to detect the protein expression levels of AKT, p-AKT, mTOR, p-mTOR, Beclin-1, p62, LC3-I, and LC3-II to evaluate the influence of SXSM on autophagy and its mechanism. These results demonstrated that, when compared with the CON group, the expression levels of p-AKT and p-mTOR in the AngII group were significantly increased. Meanwhile, the expression of Beclin-1 and LC3-II/LC3-I decreased significantly, accompanied by the consumption decrease of the autophagy substrate p62, suggesting that AKT/mTOR phosphorylation of NIH-3T3 cell line was activated while the autophagy activity was inhibited. However, SXSM could significantly reduce the overexpression of p-AKT and p-mTOR induced by AngII, and the increased expression of Beclin-1 and LC3-II/LC3-I was accompanied by the increased consumption of the autophagy substrate p62. Therefore, SXSM could enhance the autophagy activity by inhibiting the phosphorylation of the AKT/mTOR signaling pathway, and AKT phosphorylation agonist SC79 reversed the effect of SXSM (Figure 6(a)). Quantitative analysis revealed statistical significance among the CON, AngII, SXSM, and SC79 groups (Figure 6(b)). These results demonstrated that the hyperphosphorylation of the Akt/mTOR signaling pathway inhibited the level of autophagy and that SXSM inhibited the phosphorylation of the Akt/mTOR signaling pathway induced by AngII so as to activate autophagy, thereby exerting a protective effect.

## 4. Discussion

Sinoatrial node fibrosis is an important endogenous factor leading to the development of SSS, which can be mainly related to the increased secretion of AngII caused by the activation of the RAAS system. AngII promoted the occurrence and development of SSS by mediating the fibrosis and apoptosis of SAN cells [7, 8]. In addition, the degenerative fibrosis of SAN caused by aging is an important reason for SSS development [29]. Therefore, in order to build a reasonable SSS model, we employed the method of slowly pumping AngII with a micro-osmotic pump. *In vivo* studies revealed that AngII could successfully induce the heart rate decrease and SAN fibrosis in mice. Meanwhile, the remarkable deposition of ECM indicated that AngII could successfully induce the transformation of fibroblasts into myofibroblasts with its activated phenotype. These results support that our experimental method is feasible and that our mouse model could successfully simulate SSS in humans. We found that SXSM treatment could significantly improve the heart rate decline and SAN fibrosis in mice, while significantly inhibiting the activation and transformation of fibroblasts. It is therefore suggested that SXSM improved the function of SAN by attenuating SAN fibrosis in SSS mice.

Some past studies have reported that autophagy plays an important role in the process of cardiac fibrosis and that it may be involved in anti-fibrosis to play a cardioprotective role [30–32]. The literature revealed that autophagy is an indispensable defense mechanism involved in the pathogenesis of myocardial fibrosis [33]. In order to explore whether the mechanism of SXSM attenuating SAN fibrosis was related to autophagy, we used NIH-3T3 mouse fibroblasts to simulate SAN fibroblasts *in vitro* experiments. MDC staining and Western blotting results showed that the autophagy activity of NIH-3T3 cells administered by AngII decreased significantly, accompanied by a decrease in the number of autophagosomes. Meanwhile, the expression of *α*-SMA and the deposition of ECM were detected by immunofluorescence staining, indicating that AngII may promote the activation and transformation of fibroblasts by inhibiting the autophagy level of NIH-3T3 cells. Therefore, activating autophagy may be an important approach to resist fibrosis. We thus speculated that SXSM may attenuate fibrosis by activating the cell autophagy level. To prove this conjecture, we added SXSM when treating NIH-3T3 cells with AngII and found that, after SXSM treatment, the autophagy level of NIH-3T3 cells increased while the expression of *α*-SMA and ECM protein decreased significantly. This part of the experiment thus proves that SXSM could regulate the expression of fibrotic proteins such as *α*-SMA and ECM (including fibronectin and collagen-I) by activating autophagy at the cellular level, thereby inhibiting the transformation of fibroblasts into myofibroblasts with their activated phenotype.

Several past studies have reported that a variety of signaling pathways are involved in the regulation of autophagy, among which the Akt/mTOR signaling pathway plays an important role, mainly in the baseline regulation and stress regulation of autophagy [18, 19]. Western blotting results also showed that AngII could upregulate the phosphorylation level of the AKT/mTOR signaling pathway in NIH-3T3 cells while simultaneously decreasing the autophagy activity, thereby indicating that AngII possibly inhibits autophagy by activating the phosphorylation of the AKT/mTOR signaling pathway. In order to explore whether SXSM could activate autophagy by inhibiting the phosphorylation level of the AKT/mTOR signaling pathway, we added SXSM when treating NIH-3T3 cells with AngII. We found that the phosphorylation level of the AKT/mTOR signaling pathway was inhibited and that the autophagy activity was enhanced after SXSM treatment. For further demonstration, we provided AKT phosphorylation agonist SC79 on the basis of SXSM treatment and found that the therapeutic effect of SXSM was blocked by SC79 through MDC staining, immunofluorescence staining, and Western blotting. This part of the experiment proved that SXSM could regulate autophagy by regulating the phosphorylation level of the AKT/mTOR signaling pathway.

## 5. Conclusion

SXSM may activate autophagy by inhibiting the phosphorylation of the AKT/mTOR signaling pathway, which is followed by the inhibition of the activation of fibroblasts and excessive secretion of ECM induced by AngII, thereby improving SAN fibrosis and protecting the SAN.

## Figures and Tables

**Figure 1:** SXSM improved the function of the SAN as well as increased the heart rate of the SSS mice. (a)The resting heart rate of each group of mice (125 ms/Div). (b)The statistical analysis of the heart rate in each mice group. (c)The statistical analysis of the R-R interval of the electrocardiogram in each group of mice. ^*∗∗*^*P* < 0.01 vs. SSS. SHAM: Sham-operation group. SSS: sick sinus syndrome model group. SXSM: Shenxian-Shengmai oral liquid treatment group.

**Figure 2:** SXSM attenuates SAN fibrosis in SSS mice. (a)Masson's trichrome staining of the SAN area of mice in each group. (b)Immunofluorescence staining of fibronectin and collagen-I in the SAN area of mice in each group. (c)Statistical analysis of the collagen volume fraction in the SAN area of mice in each group. (d)The results of the statistical analysis of the average optical density of fibronectin and collagen-I in the SAN area of mice in each group. ^*∗∗*^*P* < 0.01 vs. SSS. SHAM: sham-operation group. SSS: sick sinus syndrome model group. SXSM: Shenxian-Shengmai oral liquid treatment group.

**Figure 3:** Experimental results of CCK-8 assay. The control group cell viability was set to 100%. This analysis showed that SXSM did not induce cytotoxicity at the 10 mL/L concentration treatment for 48 h and demonstrated the most obvious effect on the NIH-3T3 cell line at the concentration of 1 mL/L.

**Figure 4:** SXSM improved the fibrosis of NIH-3T3 cells induced by AngII, and this effect could be blocked by SC79. (a)Immunofluorescence staining of NIH-3T3 cell fibrosis marker protein. (b)Statistical analysis of collagen-I average optical density. (c)Statistical analysis of fibronectin average optical density. (d)Statistical analysis of the *α*-SMA average optical density. ^##^*P* < 0.01 vs. AngII; ^*∗∗*^*P* < 0.01 vs. SXSM. CON: control group cells. Ang II: cells treated with AngII. SXSM: cells treated with AngII and SXSM. SC79: cells treated with AngII, SXSM, and SC79. AngII: angiotensin II; SXSM: Shenxian-Shengmai oral liquid; SC79: AKT phosphorylation agonist.

**Figure 5:** SXSM attenuated the autophagy inhibition of AngII on NIH-3T3 cells; this effect could be blocked by SC79. (a)MDC staining of NIH-3T3 cells. (b)Transmission electron microscopy observation of autophagosomes of NIH-3T3 cells. Scale bar: 5 *μ*m, 2 *μ*m. (c)Statistical analysis of MDC staining of NIH-3T3 cells.(d)Statistical analysis the of number of autophagosomes. ^#^*P* < 0.05 vs. AngII, ^##^*P* < 0.01 vs. AngII; and ^*∗∗*^*P* < 0.01 vs. SXSM. CON: control group cells. Ang II: cells treated with AngII. SXSM: cells treated with AngII and SXSM. SC79: cells treated with AngII, SXSM, and SC79. AngII: angiotensin II; SXSM: Shenxian-Shengmai oral liquid; SC79: AKT phosphorylation agonist.

**Figure 6:** Protein assay of the Akt/mTOR signaling pathway and autophagy in NIH-3T3 cells. (a)Western blotting was applied to detect the expression of AKT, p-AKT, mTOR, p-mTOR, Beclin-1, p62, and LC3-II/LC3-I; (b)Quantitative analysis of the Western blotting results (a) ^#^*P* < 0.05 vs. AngII, ^##^*P* < 0.01 vs. AngII; ^*∗*^*P* < 0.05 vs. SXSM, and ^*∗∗*^*P* < 0.01 vs. SXSM. CON: control group cells. Ang II: cells treated with AngII. SXSM: cells treated with AngII and SXSM. SC79: cells treated with AngII, SXSM, and SC79. AngII: angiotensin II; SXSM: Shenxian-Shengmai oral liquid; SC79: AKT phosphorylation agonist.

## Data Availability

The data used to support the findings of this study are available from the corresponding author upon reasonable request.
